The article "Ferroptosis-Specific Inhibitor Ferrostatin-1 Relieves H2O2-Induced Redox Imbalance in Primary Cardiomyocytes through the Nrf2/ARE Pathway" was published in 2022. Journal: Dis Markers.

# Ferroptosis-Specific Inhibitor Ferrostatin-1 Relieves H_2_O_2_-Induced Redox Imbalance in Primary Cardiomyocytes through the Nrf2/ARE Pathway

**DOI:** 10.1155/2022/4539932

**Published:** 2022-02-22

**Authors:** Chaofeng Sun, Fang Peng, Jianfei Li, Xudong Cui, Xin Qiao, Wangliang Zhu

**Affiliations:** ^1^The First Affiliated Hospital of Xi'an Jiaotong University, Xi'an, China; ^2^Inner Mongolia Autonomous Region People's Hospital, Hohhot, China

## Abstract

**Objective:**

Ischemic heart disease (IHD) has always been the focus of attention of many researchers in cardiovascular disease, and its pathogenesis is also very complicated. Ferroptosis may be involved in the occurrence and development of IHD.

**Methods:**

First, primary cardiomyocytes were treated with H_2_O_2_ to simulate the IHD in vitro model. After pretreatment with different concentrations of ferrostatin-1, cell survival rate was detected by MTT method, cell apoptosis was detected by TUNEL staining and flow cytometry, and the expression of oxidative stress, ferroptosis, and related molecules of Nrf2/ARE pathway was detected by Western blotting (WB) and quantitative real-time polymerase chain reaction (qRT-PCR).

**Results:**

The mortality of primary cardiomyocytes in the H_2_O_2_ group was obviously increased. Ferrostatin-1 treatment can effectively inhibit cell death, improve antioxidant enzyme activity, inhibit the expression of ferroptosis-related molecules, and activate Nrf2/ARE pathway expression.

**Conclusion:**

Ferroptosis-specific inhibitor ferrostatin-1 relieves H_2_O_2_-induced redox imbalance in primary cardiomyocytes through the Nrf2/ARE pathway, inhibits ferroptosis, and thereby slows cardiomyocyte death.

## 1. Introduction

Ischemic heart disease (IHD) is the most common cause of health problems and heart failure in the world. As a common chronic disease, IHD can often cause myocardial ischemia, hypoxia, and even necrosis, posing a serious threat to human health [1]. An important pathophysiological mechanism of IHD is oxidative stress (OS) injury. In the process of OS injury, it will not only cause cell apoptosis and autophagy but also cause changes in cell energy metabolism [2–4]. In the occurrence of IHD, cardiomyocytes produce a large number of oxygen free radicals, and at the same time, the activity of antioxidant enzymes in the cells is reduced, resulting in lipid peroxidation on the cell membrane, the change of membrane permeability, and the destruction of cell function and structure and inducing the occurrence of cell death [5]. With the increase of the global aging population, IHD has become one of today's serious social problems. Therefore, the research on the pathogenesis, prevention, and treatment of IHD has profound significance.

The article "Ferroptosis-Specific Inhibitor Ferrostatin-1 Relieves H2O2-Induced Redox Imbalance in Primary Cardiomyocytes through the Nrf2/ARE Pathway" was published in 2022. Journal: Dis Markers.

In 2012, DiXOri discovered a new nonapoptotic cell death form, ferroptosis, while studying the small molecule Erastin to kill cancer cells containing the RAS mutation of the oncogene [6]. Ferroptosis is an iron-dependent unique form of cell death that involves a complex array of biochemical reactions, gene expression, and signaling. At present, the study found ferroptosis in morphology, biochemistry, etc., is different from apoptosis, autophagy, necrosis, etc., the process does not depend on the classic apoptosis pathway, at the same time, it is also not affected by other cell death inhibitor, its performance of the typical morphological features of mitochondria in cells becomes smaller, but the double membrane density increases, and its metabolism process involves the increase of cytoplasmic ROS and lipid ROS [7, 8]. At present, the discovery and research of ferroptosis are mainly related to tumor cell death, but it is not clear how it relates to noncancerous cells.

Ferrostatin-1 (Fer-1) is a synthetic antioxidant. It inhibits iron death more effectively than phenolic antioxidants. Fer-1 is the first ferroptosis inhibitor and is widely used in vitro and in vivo experiments [9]. The antiferroptosis function of Fer-1 mainly depends on the inhibition of lipid peroxidation.

Recent studies have shown that healthy cells are also affected by a similar “iron death” mechanism, and the key to this process is the glutathione peroxidase 4 (GPX4) protein [10]. GPX4 is the only known enzyme that can effectively reduce lipid peroxidation in biofilms. Studies have shown that silencing or overexpressing the GPX4 gene can obviously change the sensitivity of cells to ferroptosis inducer FINS (Erastin, etc.). By inhibiting System xc-blocking cystine uptake and depleting cell glutathione (GSH), Erastin leads to the inactivation of GPX4, resulting in an increase in cytoplasmic ROS and lipid ROS, which ultimately triggers ferroptosis [11]. Therefore, the occurrence of ferroptosis has a similar mechanism to the increase of oxygen radicals and the decrease of antioxidant enzyme activity in the known pathogenesis of IHD, both of which are related to ROS.

There are few researches of ferroptosis in IHD. We hypothesized that ferroptosis could be regulated to inhibit cardiomyocyte damage during the occurrence of IHD.

## 2. Materials and Methods

### 2.1. Primary Cardiomyocyte Extraction

Newborn specific pathogen free (SPF) grade Sprague Dawley (SD) rats, 1 to 3 days, male and female, with a body weight of about 5 to 6 g, were provided by Henan Animal Experiment Center. The apex of the suckling mouse was removed under aseptic conditions, it was washed with phosphate-buffered saline (PBS, Jia May, Shanghai, China) at 4°C for three times, and then, it was cut into a tissue block of about 1 mm^3^ in size and mixed with 0.08% trypsin-containing cardiomyocyte digestion solution (Jia May, Shanghai, China). Then, the tissue was transferred to a glass bottle and incubated in a 37°C water bath for 6 min. It was precipitated naturally, and the supernatant was discarded. The digestion was repeated about 7-8 times in the same way until the tissue block became white and translucent. The supernatant after each natural precipitation was mixed with an equal volume of Dulbecco's Modified Eagle Medium (DMEM; Life Technology, Wuhan, China) medium containing 20% fetal bovine serum (FBS; Life Technology, Wuhan, China) and centrifuged at 1000 r/min for 5 min. Then the supernatant was discarded, and the cells were cultured with DMEM containing 10% FBS in a 37°C, 5% CO_2_ incubator for differential adherent culture. After 90 min, we drew the cell suspension, and the cells were centrifuged at 1000 r/min for 5 min. Then, the supernatant was discarded, and the cells were mixed with the complete medium to make a cell suspension. The cell concentration was adjusted to 4 × 10^5^/mL with complete medium and added to 0.1 mmol/L Brdu solution (Life Technology, Wuhan, China) to inhibit the proliferation of fibroblasts. After 48 hours of culture, the supernatant was discarded. DMEM medium was cultured simultaneously for 24 h.

The article "Ferroptosis-Specific Inhibitor Ferrostatin-1 Relieves H2O2-Induced Redox Imbalance in Primary Cardiomyocytes through the Nrf2/ARE Pathway" was published in 2022. Journal: Dis Markers.

### 2.2. Cell Grouping and Processing

The primary cardiomyocytes were seeded in 6-well plates, and the cells were divided into 4 groups: control, H_2_O_2_ (Jia May, Shanghai, China) treatment, 3 *μ*M ferrostatin-1+200 *μ*M H_2_O_2_ treatment, and 12 *μ*M ferrostatin-1+200 *μ*M H_2_O_2_ treatment. Ferrostatin-1 powder (Med Chem Express, Shanghai, China) was dissolved in dimethyl sulfoxide (DMSO) (Jia May, Shanghai, China) and formulated into a solution with a concentration of 50 mM and stored at -80°C until use. When the experiment was used, the medium was diluted to the required working concentration.

### 2.3. MTT (3-(4,5-Dimethylthiazol-2-yl)-2,5-Diphenyl Tetrazolium Bromide)

The primary cardiomyocytes were seeded in 96-well plates at approximately 2 × 10^4^ cells per well. The experiment was set up with 6 multiple wells, and a normal control group and a blank control group were set. After cells were incubated in a 37°C, 5% CO_2_ incubator overnight, the original culture solution was discarded. The normal control group was replaced with complete medium. The blank control group was added with equal volume of phosphate-buffered saline (PBS). The H_2_O_2_ group was added with 200 *μ*M H_2_O_2_. The ferrostatin-1 group was added with different concentrations (3, 6, and 12 *μ*M) of ferrostatin-1 before adding H_2_O_2_. After 12 hours of cocultivation, 5 mg/mL of 20 *μ*L MTT solution (Jian Cheng, Nanjing, China) was added to each well. Four hours later, the supernatant was discarded, 150 *μ*L DMSO was added to each well, and it was shaken steadily for 10 min. It was placed on the enzyme-linked immunoassay detector (Rongjin, Shenzhen, China), the optical density value (OD value) of each well was detected at a wavelength of 490 nm, and the experiment was repeated 3 times.

The article "Ferroptosis-Specific Inhibitor Ferrostatin-1 Relieves H2O2-Induced Redox Imbalance in Primary Cardiomyocytes through the Nrf2/ARE Pathway" was published in 2022. Journal: Dis Markers.

### 2.4. Lactic Dehydrogenase (LDH) Kit Detection

According to the experimental grouping, the supernatant solution of each group was collected, and the configured working solution (Thermo Fisher Scientific, Waltham, MA, USA) was added and was reacted in the water bath at 37°C for 15 minutes each time. Finally, 0.4 mol/L NaOH solution was added, and the absorbance of each group was determined by enzyme-linked immunoassay detector with the wavelength of 450 nm after oscillating and mixing.

### 2.5. Superoxide Dismutase (SOD) Kit Detection

According to the experimental grouping, we collected the supernatant solution of each group, added the configured working solution (Thermo Fisher Scientific, Waltham, MA, USA), and reacted in the water bath at 37°C for 20 minutes. After oscillating and mixing, the absorbance of each group was determined by enzyme-linked immunoassay detector at a wavelength of 450 nm.

### 2.6. GSH Kit Detection

We collected the cells and suck up the supernatant. The protein removal reagent S solution (Thermo Fisher Scientific, Waltham, MA, USA) was added and vortexed fully and evenly. Then, the samples were freeze-thawed rapidly twice by liquid nitrogen and 37°C water baths. Next, the samples were centrifuged at 4°C at 10000 r/min for 10 min. The supernatant was used for the determination of total GSH, and the contents of each group were compared.

### 2.7. Intracellular MDC Levels Were Detected by Flow Cytometry

The primary cardiomyocytes were inoculated with 2 × 10^5^ per well in a 6-well plate, and the cells were cultured in an incubator at 37°C for 24 hours. After the cells were treated as above, 1 ml of MDC dye solution (Jian Cheng, Nanjing, China) with final concentration of 50 *μ*M was added to each cell, and the cells were incubated in an incubator in dark for 30 minutes. After washing with PBS for 3 times, flow cytometry (Becton Dickinson, Heidelberg, Germany) was used for detection.

### 2.8. GPX Kit Detection

The experiment was divided into control group, H_2_O_2_ group, and 12 *μ*M ferrostatin-1 group. The test buffer, cell sample, and GPX test fluid (Thermo Fisher Scientific, Waltham, MA, USA) were added to the 96-well plate according to the requirements of the kit. After the oscillation mixing, the absorbance of each group was measured by enzyme-linked immunoassay detector at the wavelength of 340 nm, and then, the absorbance of each group was detected again every 2 min to calculate the GPX activity.

The article "Ferroptosis-Specific Inhibitor Ferrostatin-1 Relieves H2O2-Induced Redox Imbalance in Primary Cardiomyocytes through the Nrf2/ARE Pathway" was published in 2022. Journal: Dis Markers.

### 2.9. Intracellular ROS Levels Were Detected by Flow Cytometry

The cells were inoculated on a 6-well culture plate. After 24 hours of dosing and culture, the cells were digested with trypsin and centrifuged at 1500 r/min for 5 minutes, and cells of each group were collected. The cells were resuspended in DCFH-DA (Jian Cheng, Nanjing, China) serum-free medium with a final concentration of 10 *μ*M, mixed by pipetting, and incubated for 20 minutes. The cells were washed 3 times with fresh medium to fully remove the DCFH-DA. The flow cytometer detects fluorescence intensity at an excitation wavelength of 488 nm and an emission wavelength of 525 nm.

### 2.10. Immunofluorescence Staining

Cells in the logarithmic growth stage were inoculated in 6-well plates with 2 × 10^5^ cells per well, and 2 mL fresh medium was added to each well for overnight culture. After culture for 24 hours, the medium was discarded and washed twice with precooled PBS at 4°C. 1 mL of 2% paraformaldehyde was gently added to each well for fixation. After 15 minutes, the paraformaldehyde solution was discarded, 1 mL PBS was added into each well to wash the cells, and then, the diluted primary anti-SOD1 (Abcam, Cambridge, MA, USA, Rabbit, 1 : 500) was added, and it was incubated overnight at 4°C. The next day, 1 mL PBS was added to each hole and washed twice. Second antibody was added and incubated at room temperature for 1 hour. Finally, 4′,6-diamidino-2-phenylindole (DAPI) dye solution (Thermo Fisher Scientific, Waltham, MA, USA) of 1 mL/well was added, and the cells were kept out of light for 10 minutes at room temperature. Then, the cells were lightly washed with precooled PBS and observed under an inverted fluorescence microscope (Thermo Fisher Scientific, Waltham, MA, USA).

### 2.11. TUNEL Staining

2 × 10^5^ cells of log phase-proliferated primary cardiac myocytes were inoculated into 24-well plates and cultured for 12 hours in an incubator. Then, the cells of different treatment groups were stained with TUNEL kit (Elabscience, Wuhan, China) in the dark. After DAPI staining, the results were observed under a fluorescence microscope (Sunny Optical, Zhejiang, China) and recorded.

### 2.12. Western Blot Test

The cell protein was collected by radioimmunoprecipitation assay (RIPA) protein lysate (Jia May, Shanghai, China) and centrifuged at 4°C for 10 min at 12,000 r/min. The supernatant was taken. After the protein concentration of each group was determined by bicinchoninic acid (BCA) method (Jia May, Shanghai, China), an appropriate amount of 4× protein buffer was added and boiled at 100°C for 5 min. The denatured proteins were subjected to sodium dodecyl sulphate-polyacrylamide gel electrophoresis (SDS-PAGE), film transferred, and blocked with 5% skimmed milk at room temperature for 2 hours; then, the corresponding primary antibody (SOD1, Abcam, Cambridge, MA, USA, Rabbit, 1 : 2000; SOD2, Abcam, Cambridge, MA, USA, Rabbit, 1 : 2000; FP1, Abcam, Cambridge, MA, USA, Mouse, 1 : 3000; Ptgs2, Abcam, Cambridge, MA, USA, Mouse, 1 : 2000; Nrf2, Abcam, Cambridge, MA, USA, Rabbit, 1 : 1000; HO-1, Abcam, Cambridge, MA, USA, Rabbit, 1 : 2000; GPX4, Abcam, Cambridge, MA, USA, Mouse, 1 : 1000; and GAPDH, Proteintech, Rosemont, IL, USA, 1 : 5000) was added and incubated overnight at 4°C. Then, the corresponding secondary antibody (1 : 1000 dilution, Yifei Xue Biotechnology, Nanjing, China) was added and incubated at room temperature for 2 h. After incubation with enhanced chemiluminescence (ECL, Elabscience, Wuhan, China) solution, it was developed on the chemiluminescence imaging system.

The article "Ferroptosis-Specific Inhibitor Ferrostatin-1 Relieves H2O2-Induced Redox Imbalance in Primary Cardiomyocytes through the Nrf2/ARE Pathway" was published in 2022. Journal: Dis Markers.

### 2.13. Total RNA Extraction and Quantitative Real-Time Polymerase Chain Reaction (qRT-PCR)

The total RNA of each group of cells was extracted according to the instructions of the RNA rapid extraction kit (Thermo Fisher Scientific, Waltham, MA, USA). The ultraviolet spectrophotometer (Becton Dickinson, Heidelberg, Germany) was used to determine the purity and concentration of RNA. The primer sequence of the target gene after reverse transcription is shown in Table 1.

### 2.14. Statistical Analysis

Statistical analysis was performed using the Prism 8.0 (GraphPad software, La Jolla, CA, USA) software. Each experiment was repeated 3 times. The experimental data was expressed as mean ± standard deviation (mean ± SD). The comparison of the two groups of data was performed by independent sample *t* test. Analysis of variance was used for comparison among multiple groups. *P* < 0.05 was considered statistically significant, and *P* < 0.01 was considered statistically significant.

## 3. Results

### 3.1. Effects of H_2_O_2_ and Ferrostatin-1 on the Survival Rate of Primary Cardiomyocytes

In order to establish the H_2_O_2_ concentration suitable for the OS injury model of primary myocardial cells, H_2_O_2_ concentration was divided into 5 groups (0 *μ*mol/L, 50 *μ*mol/L, 100 *μ*mol/L, 200 *μ*mol/L, and 400 *μ*mol/L). After 4 hours of H_2_O_2_ treatment, the survival rate of each group was detected by MTT kit (Figure 1(a)). The results showed that compared with the control group, with the increase of H_2_O_2_ concentration, the cell survival rate gradually decreased. At the same time, we examined the effect of different ferrostatin-1 concentrations on the survival rate of primary cardiomyocytes using the MTT kit (Figure 1(b)). The results showed that after ferrostatin-1 was applied to primary cardiomyocytes at a concentration range of 3 *μ*M–12 *μ*M for 12 hours, there was no significant change in cell survival compared with the normal group, indicating that ferrostatin-1 had no significant effect on the growth of primary cardiomyocytes at this dose range. Next, we pretreated the cells with ferrostatin-1 for 12 hours, then added 200 *μ*mol/L H_2_O_2_ for 2 hours, and tested the cell survival rate with the MTT kit (Figure 1(c)). The results show that 3-12 *μ*M ferrostatin-1 has a protective effect on primary cardiomyocytes injured by H_2_O_2_, and its protective effect was concentration-dependent. Among them, 12 *μ*M ferrostatin-1 can obviously inhibit H_2_O_2_-induced cell death. At the same time, in order to detect the damage degree of H_2_O_2_ to cells and cell membrane, we detected the LDH activity in the cell supernatant and found that the LDH activity in the cell supernatant after the treatment of 12 *μ*M ferrostatin-1 alone had no significant change compared with the control group (Figure 1(d)). After the injury of 200 *μ*mol/L H_2_O_2_, the LDH activity in the cell supernatant obviously increased. On the contrary, the LDH activity in the supernatant of the ferrostatin-1 group was lower than that of the H_2_O_2_ group, and there was a significant difference between the H_2_O_2_ group and the ferrostatin-1 group at the dose of 12 *μ*M, indicating that ferrostatin-1 could obviously inhibit the LDH leakage of H_2_O_2_-damaged primary cardiomyocytes.

The article "Ferroptosis-Specific Inhibitor Ferrostatin-1 Relieves H2O2-Induced Redox Imbalance in Primary Cardiomyocytes through the Nrf2/ARE Pathway" was published in 2022. Journal: Dis Markers.

### 3.2. Ferrostatin-1 Inhibited H_2_O_2_-Induced OS in Primary Cardiomyocytes

In order to detect the degree of redox imbalance in primary cardiomyocytes, we detected intracellular ROS levels and found that the ROS level in the 200 *μ*M H_2_O_2_ group increased, while in the 3 *μ*M and 12 *μ*M ferrostatin-1 groups, ROS level decreased obviously and was dose-dependent (Figure 2(a)). At the same time, we detected the activity of GSH and SOD in the cell supernatant and found that 3 *μ*M and 12 *μ*M ferrostatin-1 can inhibit the decrease of GSH and SOD activity caused by H_2_O_2_ (Figures 2(b) and 2(c)). Next, we detected the expression of SOD1 and SOD2 by WB and PCR (Figures 2(d)–2(f)). As a result, it was found that the expression of SOD1 and SOD2 in the H_2_O_2_ group was obviously reduced, while ferrostatin-1 can effectively promote the increase of SOD1 and SOD2 expression, and the 12 *μ*M ferrostatin-1 group was more significant. Then, we detected the expression of SOD1 in primary cardiomyocytes by immunofluorescence staining, and the results obtained were similar to the former (Figure 2(g)).

### 3.3. Ferrostatin-1 Inhibited H_2_O_2_-Induced Ferroptosis in Primary Cardiomyocytes

Studies have confirmed that ferroportin1 (FP1) plays an important role in the process of cellular iron circulation [12]. WB results showed that compared with the control group, FP1 protein expression in the H_2_O_2_ group obviously decreased, while compared with the H_2_O_2_ group, FP1 protein expression in the 12 *μ*M ferrostatin-1 group was obviously upregulated, showing a significant difference, while in the 3 *μ*M ferrostatin-1 group, there was no significant difference (Figure 3(a)). Similar results were obtained by qRT-PCR (Figure 3(b)). In order to further prove the occurrence and situation of ferroptosis in the primary cardiomyocyte model of H_2_O_2_ injury, we detected the level of prostaglandin peroxidase 2 (Ptgs2) protein (Figure 3(c)). Compared with the control group, the expression of Ptgs2 in the H_2_O_2_ group was obviously increased and there was a significant difference; after pretreatment with ferrostatin-1, the expression of Ptgs2 protein could be obviously reduced. At the same time, we also detected the expression of Ptgs2 mRNA (Figure 3(d)). The expression of Ptgs2 mRNA in the H_2_O_2_ group was higher than that in the control group, and the difference was statistically significant; compared with the H_2_O_2_ group, with the increase in the concentration of ferrostatin-1, the expression level of Ptgs2 mRNA decreased. This result was consistent with the results of protein level experiments, suggesting that ferrostatin-1 can inhibit the occurrence of ferroptosis induced by H_2_O_2_ in primary cardiomyocytes. At the same time, in order to quantitatively analyze the level of cell autophagy, we used flow cytometry to detect monodansylcadaverine (MDC) fluorescence intensity (Figure 3(e)). Studies confirm that MDC is commonly considered a specific marker for detecting autophagosome formation [13]. And our results showed that compared with the control group, the fluorescence intensity of the H_2_O_2_ group increased, suggesting that the model cells do exist autophagy; adding different doses of inhibitor ferrostatin-1, compared with the H_2_O_2_ group, the average fluorescence intensity did not obviously weaken. It suggests that there may be weak autophagy in the cell, but ferrostatin-1 was not a protective effect by inhibiting autophagy. In addition, observation of TUNEL staining by fluorescence microscopy showed that the number of positive cells in the H_2_O_2_ group was significantly higher than that in the control group, while in the ferrostatin-1 group, the inhibitory effect of different concentrations of ferrostatin-1 on the number of positive cells was not obvious (Figure 3(f)).

The article "Ferroptosis-Specific Inhibitor Ferrostatin-1 Relieves H2O2-Induced Redox Imbalance in Primary Cardiomyocytes through the Nrf2/ARE Pathway" was published in 2022. Journal: Dis Markers.

### 3.4. Nrf2/ARE Pathway Was Involved in H_2_O_2_-Induced Ferroptosis of Primary Cardiomyocytes

The Nrf2/ARE pathway is currently widely regarded as a defensive molecular pathway for the body to resist oxidative and chemical stimuli in the internal and external environment [14]. Nrf2 can regulate the oxidation and anti-inflammatory proteins of many endogenous genes in cells [15, 16], such as HO-1 and GPX4. WB results showed that compared with the control group, the levels of Nrf2, HO-1, and GPX4 protein in the H_2_O_2_ group were decreased, and there was a significant difference (Figure 4(a)). After pretreatment with 12 *μ*M ferrostatin-1, it can obviously promote the upregulation of Nrf2, HO-1, and GPX4 protein expression. At the same time, qRT-PCR also obtained similar results (Figures 4(b)–4(d)). Next, we tested the activity of GPX in the cell supernatant, and the results showed that the GPX level of the H_2_O_2_ group cells was obviously reduced compared to the control group (Figure 4(e)). The results indicated that H_2_O_2_ induced cell ferroptosis by reducing the level of GPX. Compared with the H_2_O_2_ group, the 12 *μ*M ferrostatin-1 group had obviously higher GPX levels. The above results suggest that ferrostatin-1 can reduce the damage of H_2_O_2_ on primary cardiomyocytes, and its mechanism may be related to the upregulation of Nrf2, HO-1, and GPX4 expression and improvement of cell antioxidant capacity.

## 4. Discussion

Ferroptosis is a cell death method discovered when the small molecule substance elastin kills cancer cells containing the RAS mutation of the oncogene [17]. At present, the research of ferroptosis is only in the initial stage, mainly involving in the research of antitumor. The study found that the use of antitumor drugs such as sorafinib to induce ferroptosis in cancer cells suggests that ferroptosis can be used as a new target for antitumor therapy [18]. However, whether this type of cell death is involved in other diseases besides tumors and whether there is an accurate detection method to confirm its existence, these series of problems need to be studied and confirmed.

In this study, in order to study the relationship between the primary cardiomyocyte death caused by H_2_O_2_ and ferroptosis, first, we found that ferroptosis-specific inhibitor ferrostatin-1 can obviously improve the primary cardiomyocyte status and reduce cell death. Cell death is a complicated process, in which different forms of death such as autophagy and apoptosis coexist [19]. In this experiment, by detecting different indicators such as MDC and TUNEL, it was confirmed that the form of cell death can coexist in the process of primary myocardial cell injury. In this experiment, compared with the model group, the fluorescence intensity of MDC in the ferrostatin-1 group did not increase and the number of TUNEL positive cells did not increase in the ferrostatin-1 group, but the cell viability was obviously improved, indicating that ferrostatin-1 did not inhibit apoptosis, autophagy, etc.

The article "Ferroptosis-Specific Inhibitor Ferrostatin-1 Relieves H2O2-Induced Redox Imbalance in Primary Cardiomyocytes through the Nrf2/ARE Pathway" was published in 2022. Journal: Dis Markers.

Therefore, we speculate that H_2_O_2_ induces iron-related death in primary cardiomyocytes. Cell iron load is an important factor affecting ferroptosis. Studies have shown that FP1 is a transmembrane iron export protein present on the cell membrane. FP1 is an important protein that maintains the balance of iron concentration in the cell, and it plays an important role in the transfer and export of iron. The results of this experiment found that after primary cardiomyocytes treated with 200 *μ*M H_2_O_2_, the expression level of FP1 protein in the cells decreased compared with the control group, indicating that the induction of H_2_O_2_ affected the iron homeostasis of the cells. This also confirms that the cell damage caused by H_2_O_2_ is related to iron-related death. In addition, Ptgs2 is a key enzyme in the prostaglandin synthesis process. It can increase the peroxidase activity through prostaglandin and other metabolites, leading to the generation of free radicals and affecting the oxidation balance of the body. Therefore, the upregulation of Ptgs2 protein is believed to be a ferroptosis occurring in marker [20]. In view of this, we detected the Ptgs2 protein and mRNA levels, and the results showed that the Ptgs2 protein and mRNA levels of the model group were upregulated simultaneously.

The results of this series further confirmed that H_2_O_2_ induced primary cardiomyocyte death mainly due to the occurrence of ferroptosis. Therefore, further in-depth study of ferroptosis exploring the mechanism of its occurrence in myocardial cell injury model is needed. The detection of ferroptosis presence of accurate indicators and methods will have important significance for the treatment of IHD.

## 5. Conclusion

Ferroptosis-specific inhibitor ferrostatin-1 alleviates H_2_O_2_-induced redox imbalance in primary cardiomyocytes through the Nrf2/ARE pathway, inhibits ferroptosis, and thus slows cardiomyocyte death. This provides a new basis for clinical treatment of IHD.

The article "Ferroptosis-Specific Inhibitor Ferrostatin-1 Relieves H2O2-Induced Redox Imbalance in Primary Cardiomyocytes through the Nrf2/ARE Pathway" was published in 2022. Journal: Dis Markers.

## Figures and Tables

**Figure 1:** Effects of H_2_O_2_ and ferrostatin-1 on the survival rate of primary cardiomyocytes. (a) The effect of H_2_O_2_ on cell viability was detected by MTT (“∗” indicates statistical difference from the 0 *μ*M H_2_O_2_ group, *P* < 0.05; “∗” indicates statistical difference from the 0 *μ*M H_2_O_2_ group, *P* < 0.01). (b) The effect of ferrostatin-1 on cell viability was detected by MTT. (c) The effect of ferrostatin-1 on H_2_O_2_-induced cell viability was detected by MTT. (d) LDH activity was detected by kit (“∗∗” indicates statistical difference from the control group, *P* < 0.01; “#” indicates statistical difference from the H_2_O_2_ group, *P* < 0.05; “##” indicates statistical difference from the H_2_O_2_ group, *P* < 0.05).

**Figure 2:** Ferrostatin-1 inhibited H_2_O_2_-induced oxidative stress in primary cardiomyocytes. (a) Intracellular ROS levels were detected by flow cytometry. (b) GSH activity was detected by kit. (c) SOD activity was detected by kit. (d) SOD1 and SOD2 protein level was detected by WB. (e) SOD1 mRNA level was detected by qRT-PCR. (f) SOD2 mRNA level was detected by qRT-PCR. (g) The expression of SOD1 was detected by immunofluorescence staining (“∗” indicates statistical difference from the control group, *P* < 0.05; “∗∗” indicates statistical difference from the control group, *P* < 0.01; “#” indicates statistical difference from the H_2_O_2_ group, *P* < 0.05; “##” indicates statistical difference from the H_2_O_2_ group, *P* < 0.05).

**Figure 3:** Ferrostatin-1 inhibited H_2_O_2_-induced ferroptosis in primary cardiomyocytes. (a) FP1 protein level was detected by WB. (b) FP1 mRNA level was detected by qRT-PCR. (c) Ptgs2 protein level was detected by WB. (d) Ptgs2 mRNA level was detected by qRT-PCR. (e) MDC fluorescence intensity was detected by flow cytometry. (f) The cell apoptosis was detected by TUNEL staining (“∗∗” indicates statistical difference from the control group, *P* < 0.01; “#” indicates statistical difference from the H_2_O_2_ group, *P* < 0.05; “##” indicates statistical difference from the H_2_O_2_ group, *P* < 0.05).

**Figure 4:** Nrf2/ARE pathway was involved in H_2_O_2_-induced ferroptosis of primary cardiomyocytes. (a) Nrf2, HO-1, and GPX4 protein level was detected by WB. (b) Nrf2 mRNA level was detected by qRT-PCR. (c) HO-1 mRNA level was detected by qRT-PCR. (d) GPX4 mRNA level was detected by qRT-PCR. (e) GPX activity was detected by kit (“∗∗” indicates statistical difference from the control group, *P* < 0.01; “#” indicates statistical difference from the H_2_O_2_ group, *P* < 0.05; “##” indicates statistical difference from the H_2_O_2_ group, *P* < 0.05).

The article "Ferroptosis-Specific Inhibitor Ferrostatin-1 Relieves H2O2-Induced Redox Imbalance in Primary Cardiomyocytes through the Nrf2/ARE Pathway" was published in 2022. Journal: Dis Markers.

**Table 1:** qRT-PCR primers.

Gene name	Forward (5′>3′)	Reverse (5′>3′)
FP1	CAACCCGCTCCCATAAG	GGCAAACAACAACAGCAA
Ptgs2	TTCAACACACTCTATCACTGGC	AGAAGCGTTTGCGGTACTCAT
GPX4	TTCTCAGCCAAGGACATCG	CACTCAGCATATCGGGCAT
Nrf2	GATGGACTTGGAGTTGCC	CCTTCTGGAGTTGCTCTTG
HO-1	ACAGCCCCACCAAGTTC	GGCGGTCTTAGCCTCTTC
SOD1	GGTGAACCAGTTGTGTTGTC	CCGTCCTTTCCAGCAGTC
SOD2	CAGACCTGCCTTACGACTATGG	CTCGGTGGCGTTGAGATTGTT
GAPDH	ACAACTTTGGTATCGTGGAAGG	GCCATCACGCCACAGTTTC

qRT-PCR: quantitative reverse-transcription polymerase chain reaction.

## Data Availability

The datasets used and analyzed during the current study are available from the corresponding author on reasonable request.
